# Detection of Viral Citrullinated Peptide Antibodies Directed Against EBV or VCP: In Early Rheumatoid Arthritis Patients of Indian Origin

**DOI:** 10.4103/0974-2727.72158

**Published:** 2010

**Authors:** Sudha S Deo, Rashmi R Shetty, Kejal J Mistry, Arun R Chogle

**Affiliations:** 1 Sir. H.N. Medical Research Society; Raja Ram Mohan Roy Road, Girgaum, Mumbai – 400 004, India; 2 Sir. H.N. Hospital and Research Centre, Raja Ram Mohan Roy Road, Girgaum, Mumbai – 400 004, India

**Keywords:** Anti-viral citrullinated peptides/antibodies, ERA, EBNA-1, ELISA

## Abstract

**Aim:**

Study was undertaken to analyze the frequency of anti-viral citrullinated peptide (anti-VCP) antibodies in sera from patients with early rheumatoid arthritis (ERA).

**Materials and Methods:**

Viral citrullinated peptide (VCP) and Epstein-Barr nuclear antigen (EBNA-1) peptide were commercially prepared and antibodies to these were determined in 25 patients of ERA, 40 disease control patients constituting 25 rheumatoid arthritis (RA), 7 systemic lupus erythematosus (SLE), 2 scleroderma, 1 spondyloarthritis (SpA), 1 juvenile rheumatoid arthritis (JRA), 1 osteoarthritis (OA), 1 psoriatic arthritis (PsA), 1 undifferentiated arthritis (UA), and 1 gout and 25 healthy controls (HCs) were taken for comparison. In-house ELISA was established for both the antibodies while cyclic citrullinated peptide (CCP) antibody was detected by commercial ELISA kit.

**Results:**

Significant increase in VCP antibody by ERA and disease controls than healthy normal was observed. VCP IgM antibody was significantly increased in RA patients than HC. The presence of VCP antibody signifies a good marker for ERA. We observed significant difference in the VCP IgG and IgM antibody when compared to EBNA-1. In-house ELISA established for EBNA-1 and VCP antibodies showed low sensitivity but 96% specificity.

**Conclusions:**

We observed that sera from early RA patients reacted to the deiminated protein encoded by Epstain Barr Virus (EBV). Thus a possible role of virus in inducing an anti-citrullinated peptide antibody (ACPA) response reveals viral etiology in this disease.

## INTRODUCTION

The present study was undertaken to detect the prevalence and the association of anti-VCP antibodies in Early Rheumatoid Arthritis (ERA) patients and compare the efficacy of these antibodies.

The notion stating that microbial species including bacteria, viruses, and other parasites represent the main stimuli for the initiation as well as sustenance of immune responses in a genetically susceptible individual has long been predicted and has been the central force for the cause of autoimmune disease research. This has led to the understanding of the infectious agent as the etiological agent in the cause of initiation of the pathogenesis of RA.

The actual mechanisms initiating these reactions are still not known. Mechanisms by which infectious agents may initiate RA and/or autoimmunity include molecular mimicry and epitope spreading. Molecular mimicry can be initiated when lingering autoreactive T cells become activated by peptides from infecting organisms that bear similar structure and/or amino acid sequence to that of same host peptide, i.e. proteins/peptides that share a similar molecular structure to that of host tissue peptides, and which therefore can perpetuate inappropriate immune reactions to self.[1] Recent studies suggest that autoantibodies to citrullinated proteins provide a useful and quite specific diagnostic indicator for RA. The anti-CCP antibody is present in approximately 80% of RA patients and is quite specific for the disorder. Moreover, this autoantibody is detected in less than 1% of healthy individuals; it can even appear before RA is clinically evident and detectable.[2]

Thus RA-specific antibodies recognize different deiminated proteins of overlapping specificities that can be called as ACPA. Citrullination or deimination is a post-translational modification of amino acid arginine in a protein into amino acid citrulline by the enzyme peptidyl-arginine deiminase (PAD). A comparative evaluation of such sequences that are recognized by ACPA show that critical feature is the presence of citrulline. Cyclic-citrullinated peptide is an artificial molecule in which two serine residues in a major epitope peptide of filaggrin is converted to cysteine and the circular form is made by a disulfide bond. The first commercial anti-CCP1-used was derived from the sequence of human filaggrin as immunosorbent.

While the CCP2 is derived from a library of highly reactive peptides, this anti-CCP2 test has increased sensitivity of 82% and 98–99% specificity. Several studies have reported the prognostic ability of CCP1 test to predict the erosive progression of RA. Thus the presence of anti-CCP antibody positivity in ERA is shown to be a strong prognostic marker for the development of erosive RA. An anti-CCP2 is used in the diagnosis of radiological joint damage and progression after two years of follow-up.

The anti-CCP was specific around 98% towards filaggrin, which is expressed only in the epithelial cells and they do not target for RA autoimmune response. Because fillagrin antibodies are not detected in synovial tissue, other molecules have been proposed as biological relevant targets. Vimentin, another citrullinated protein, is also detected by inflamed synovia and recognized by anti-filaggrin antibodies (AFAs). Besides the sequences recognized by AFAs showed the presence of citrulline flanked by neutral amino acids such as glycine, serine and threonine. Similar amino acid repeats have been found in nucleic acid binding proteins, some of which are of viral origin. One of the herpes viruses is the Epstein-Barr virus (EBV), a member of the Herpesviridae family and is known to infect B lymphocytes and epithelial cells of the oropharynx.

An EBV was first implicated in the pathogenesis of RA in 1976 and 1978.[3,4] It was reported that sera from patients with RA were reactive against a nuclear antigen in EBV transforming lymphocytes. This RA nuclear antigen was determined as glucose/alanine rich repeat in EBNA-1. Antibodies against this repeat are cross-reactive with a 62-kDa protein present in the synovium of patients with RA but not in controls. Antigenic sequence similarities exist between other EBV proteins and RA-specific proteins as well. Humans with EBV infection have antibodies against the gp110 protein as well as T cells with receptors that recognize the OKRAA motif in both gp110 and HLA-DR4.

Patients with existing RA have higher levels of antibodies against several EBV-encoded proteins including VCA, early antigen (EA), EBNA-1, and EBNA-2 than do HC. Patients suffering from RA have a ten-fold increase in EBV DNA load in peripheral blood mononuclear cells compared with that of controls and have a significantly higher number of circulating EBV-infected B cells.

It is seen that EBV genome appears to be the most disseminated in an individual as it is detected more frequently than other viruses. It is the most causative agent of mononucleosis. Around more than 95% of human adults have been infected by the virus. Because of the altered immune response to EBV that causes persistence of increased cell infections and higher viral load they add as a contributing factor towards the pathogenesis of RA. One of the proteins of EBV, the EBNA-1 contains in its N-terminal region a sequence, which is characterized by glycine-arginine repeats. Thus EBNA-1 specific cells could play a role in ACPA production and anti-viral antibodies may be produced. It has been proposed that the abnormalities in the EBV-directed immune responses and the EBV viral loads whether they are a cause or a consequence of RA, still remains a mystery. Though it has potential for molecular mimicry by polyclonal activation of B cells or an EBV-specific immune response could be a trigger for the development of RA in the genetically predisposed patients.[5]

## MATERIALS AND METHODS

A total of 25 patients showing ERA with age range from 32 to 62 years, and mean age of 47 years with an M/F ratio of 2:23 and disease duration of 1–18 months were selected for our study.

### Disease controls

Of the 40 patients included, 25 were rheumatoid arthritis (RA; 21–75 years), 7 systemic lupus erythematosus (SLE; 21–23 years), 2 scleroderma (30–40 years), 1 spondylarthritis (SpA; 40 years), 1 juvenile rheumatoid arthritis (JRA; 12 years), 1 osteoarthritis (OA; 62 years), 1 psoriatic arthritis (PsA; 43 years), 1 undifferentiated arthritis (UA; 28 years), and 1 gout (53 years) were taken as disease control. Of these 40 patients, 6 males and 34 females.

### Healthy controls

Twenty five HCs from 23 to 63 years with 9 males and 16 females were included.

All the rheumatological patients were diagnosed on the basis of American College of Rheumatology (i.e., ACR) criteria. All other autoimmune patients were diagnosed according to their respective criteria. Patients with RA and all the autoimmune patients were evaluated for their systematic involvement. Besides this, the physical findings such as height, weight, blood pressure, ESR, CRP, anti-CCP, RF (IgG, IgM) test, duration of the disease, swelling, morning stiffness and fatigue were noted. The visual assessment score (VAS), health assessment score (HAQ), and short form-36 (SF-36) questionnaire was recorded.

Ethical approval was taken from the ethical committee of the hospital and informed consent was taken from each patient before the collection of their samples. The immunological *proforma*, HAQ, and SF-36 questionnaire were filled for each patient. The project was approved by Scientific Committee of our Medical Research Society.

### Method

Two synthetic peptides for EBNA-1 and VCP were manufactured commercially for our experimental purpose from Sigma (USA).

Table 1 gives the linear sequence of the two commercially prepared peptides. EBNA-1 antigen was diluted at a concentration of 2 ug/ml in phosphate-buffered saline (PBS) pH 7.2.[5] Similarly, the VCP was diluted at 5 ug/ml in PBS. Both these antigens were used for coating of the ELISA plate, 100 ul of these antigens were added to a Nunc plate and the plate was covered with a sealer to prevent evaporation and incubated overnight at 4°C. After incubation, the plate is washed three times with 300 ul of wash buffer that contains PBS and 1% Tween 20 (PBST). After which the wells were blocked with 200 ul of blocking buffer that contains 3% bovine serum albumin (BSA) dissolved in PBS. The plate is incubated for one hour at room temperature (RT). After this, patients and control serum samples are diluted 1:200 in PBS containing 1% BSA and 0.05% Tween 20. Samples are added in duplicates at 100 ul volume and incubated for 3 h at RT. The plate is then washed three times with PBST. To this is added 100 ul of anti-human IgG antibody conjugated to alkaline phosphatase. At a dilution of 1:3000 in PBST after arriving at a dilution on the checker board, the plate is then incubated for 2 h for EBNA-1 antigen used at 2 ug/ml and for 3 h for VCP containing the antigen at 5 ug/mL at RT. The plate is then washed three times with the wash buffer. To this is added 100 ul of para nitrophenyl-phosphate (pNPP) as substrate (Sigma, USA) and incubated at RT for 30 minutes. The color of the reaction will be changed from colorless to yellow after addition of the stop solution that is 3N NaOH. The optical density of the reaction was taken for each well at 405 nm. Both the peptide reactions were taken at the same wavelength. We have used two specific conjugates namely, IgG and IgM alkaline phosphate conjugates.[6]

**Table 1:** Sequences of commercially prepared peptides

No	Type	Sequence
Peptide 1	EBNA-1	GPAGPRGGGRGRGRGRGRGHNDGG
Peptide 2	VCP	GPAGPYGGGYGYGYGYGYHNDGG

Anti-RF isotypes and anti-CCP antibody were detected on all the patients and controls using a commercial ELISA kit from Quantalite Inova diagnostics (San Diego, USA).[7] The cut-off for RF being >6 IU and that of anti-CCP was >20 IU

### Statistical analysis

SPSS version 16 was used for statistical analysis of all our data. We have used the student’s *t*-test for analysis.

## RESULTS

From Table 2 it was seen that there is no significant difference in the average age, morning stiffness and fatigue score in Early RA and Established RA patients on comparison with the Normals (Healthy individuals). We found significant differences in DAS 28, I-HAQ, SF 36, ESR, CCP and the CRP markers in both early and established RA patients. Similarly, the disease control group comprising of established RA and other autoimmune patients when compared showed significant difference in these parameters showing that these parameters are specific for autoimmune diseases.

**Table 2:** Characteristics of Rheumatoid Patients and Controls

Parameters	Early RA	Disease control	Established RA	Controls	Early RA vs controls	Disease control vs controls	Established RA vs controls	Established RA vs early RA
Mean±SE	(<1yr) N=25	(>1yr) N=40	(>1yr) N=25	N= 25	*P* value	*P* value	*P* value	*P* value
Age (years)	45±1.80	43±2.14	46±2.4	46.44±2.00	0.681	1.00	1.00	0.669
Disease duration (Months)	6.26±0.97	60.73±11.38	83.8±16	NA	NA	NA	NA	0.00***
Morning stiffness (Minutes)	54±11.5	43±6.8	57.8±8.2	NA	NA	NA	NA	0.788
Fatigue (0-10 mm)	6.4±1.25	9.9±2.4	13.3±3.5	NA	NA	NA	NA	0.06
DAS28	6.2±0.27	5.5±0.3	6.1±0.26	0	0.00***	0.00***	0.00***	0.788
I-HAQ	1.35±0.1	0.99±0.1	1.16±0.13	0.17±0.08	0.00**	0.005**	0.005**	0.338
SF-36	43.6±3.8	55.2±3.8	49.96±4.47	88.9±2.79	0.00**	0.001**	0.001**	0.439
ESR (mm/hr)	59±7.5	59±6.5	70±8.25	25.7±4	0.002**	0.00***	0.00***	0.339
Anti-CCP (U/ml)	494.8±154	251.9±104	387±161.5	18±0.15	0.005**	0.031*	0.031*	0.610
CRP (mg/l)	69±14.5	62.7±14	59.9±20.72	7.5±.96	0.00**	0.016*	0.016*	0.688

* *P*<0.05;

** *P*<0.01;

*** *P*<0.001

Table 3shows the analysis of antibody to EBNA-1 and VCP in different groups. VCP and EBNA-1 ELISA assays standardized by us showed that VCP antibody (IgG and IgM) was found to be highly significant in the early RA group when compared with Normals (Healthy individuals).

**Table 3:** Analysis of antibody to EBNA 1(IgG and IgM) and VCP (IgG and IgM) in different disease conditions

Parameters	Early RA	Disease control	Established RA	Controls	Early RA vs controls	Disease control vs controls	Established RA vs controls	Established RA vs early RA
Mean ± SE	(<1yr) N=25	(>1yr) N=40	(>1 yr) N=25	N= 25	*P* value	*P* value	*P* value	*P* value
EBNA IgG	0.84±O.11	0.77±0.06	0.622±0.04	0.91±0.07	0.513	0.001**	0.091	0.091
EBNA IgM	0.53±0.08	0.5±0.05	0.509±0.06	0.41±0.06	0.313	0.23	0.858	0.858
VCP IgG	1.10±0.17	0.96±0.10	1.03±0.16	0.62±0.056	0.020*	0.035*	0.758	0.785
VCP IgM	0.95±0.97	1.27±0.09	1.15±0.11	0.62±0.064	0.013*	0.001**	0.147	0.147

+Values are represented in Mean OD of duplicates in ELISA assay

While the established RA group did not show any significant difference in VCP antibody, we can predict VCP antibody to be a specific marker for the early RA group. However, when we compared the disease controls with the HCs, both EBNA-1 and VCP (IgG and IgM) were highly significant (*P* < 0.001).

Table 4 gives the correlation analysis between EBNA-1 and VCP parameters in the early RA, the disease control and the HCs. By the Spearman’s correlation analysis, we observed that there is an association of VCP IgG antibodies with EBNA-1 IgG. Similar findings were found in VCP IgM antibodies and EBNA IgM antibodies. This clearly shows EBNA-1 contains in its N-terminal region a sequence, which is characterized by glycine-arginine repeats that could play a role in ACPA production and anti-viral antibodies may be produced.

**Table 4:** Correlation analysis between all EBNA-1 and VCP parameters in ERA = 25, Non-ERA = 40, Controls = 25

Spearman’s rho		EBNAIgG	EBNAIgM	VCPIgG	VCPIgM
EBNAIG	Correlation coefficient	1.000	-0.103	0.279**	0.070
	Sig. (2-tailed)	–	0.334	0.008	0.514
	N	90	90	90	90
EBNAIM	Correlation coefficient	-0.103	1.000	-.103	0.304**
	Sig. (2-tailed)	0.334	–	0.335	0.004	
	N	90	90	90	90
VCPIgG	Correlation coefficient	0.279**	-0.103	1.000	0.075
	Sig. (2-tailed)	0.008	0.335	–	0.482
	N	90	90	90	90
VCPIgM	Correlation coefficient	0.070	0.304**	0.075	1.000
	Sig. (2-tailed)	0.514	0.004	0.482	–
	N	90	90	90	90

** Correlation is significant at the 0.01 level (2-tailed)

Figure 1 shows the presence of viral-citrullinated antibody, standardized and detected by ELISA in our laboratory. We observed clear differences in the type of VCP antibody produced by these patients, where VCP IgG is more than VCP IgM. Similarly, there is a significant increase in the VCP produced by the early RA and disease controls than that of the healthy normal. VCP IgM antibody is a better marker than VCP IgG when compared to healthy normal. A significant number of patients (early RA and established RA) in the VCP IgM group showed higher values of antibodies as detected by in-house ELISA when it was compared to normal HC of mean + 2SD. Thus the presence of VCP antibody also can be taken as good marker for patients of RA.

**Figure 1:** Analysis of EBNA-1 (IgG and IgM) and VCP (IgG and IgM) antibodies by ELISA in different groups 0 = Early RA, 1 = Established RA, 2 = Disease control, 3 = Normal control

As we wanted to compare the diagnostic value of VCP antibody, we also studied the presence of antibody against EBNA-1. As shown in the literature that there is a presence of EBNA antibody shown by B lymphocytes. Hence, in order to study the efficacy of viral-citrullinated antibody, we tested this peptide in our in-house ELISA assay. On comparison, we observed a significant difference in the VCP IgG and VCP IgM antibody against the VCP compared to EBNA-1 peptide. Hence, we can say that VCP is a better marker than EBNA-1 viral citrullinated antibody IgM antibody and thus could be taken as significant marker for comparison between early and disease control RA patients. On comparison of this Optical Density (OD) levels between the disease control group and the HC, we can utilize the levels of antibodies against EBNA-1 antigen of the IgG type and the VCP antibody of IgG and IgM type to be specific markers distinguishing from the normal.

The in-house ELISA established by us for EBNA-1 and VCP antibodies show similar findings. It is seen that sensitivity of these assays are low and the specificity is more than 96%. EBNA-1 IgM is almost 100% specific while VCP IgG and VCP IgM show similar specificity of 96%.

Studies conducted in our laboratory showed that:

1. Viral-citrullinated antibody standardized and detected by ELISA showed clear differences in the type of VCP antibody produced by these patients wherein VCP IgG antibody produced is more than VCP IgM. There is a significant increase in the VCP produced by the early RA and disease controls than that of the healthy normal.
2. A significant number of patients (early RA and established RA) in the VCP IgM group showed higher values of antibodies on comparison with HC.
3. On comparison, we observed a significant difference in the VCP IgG and VCP IgM antibody against the VCP compared to EBNA-1 peptide. Hence, we can say that VCP is a better marker than EBNA-1.
4. Patients of early rheumatoid arthritis (ERA) show the presence of EBNA-1 (IgG) antibody, which is also associated with VCP (IgG) antibody. Similarly EBNA-1 (IgM) antibody is also associated with VCP (IgM) antibody and this is found to be statistically significant.

## DISCUSSION

From the above study we observed that sera from early RA patients also reacted to the deiminated protein encoded by EBV. Antibodies that are present in early RA and that of established RA react to EBNA-1. This suggest that since only the RA patients react to EBNA-1, there is a possibility of a role of EBV infection in the induction of the disease-specific antibodies in these patients. Since all the data is compared to HC, there is a significant association of viral antigen in response shown by the antibody. Besides this, we have also observed significant increase in the VCP antibody shown by RA patients.

It is seen from our study that RA patients showed a role of virus in inducing an ACPA response in these patients, which opens up an issue of viral etiology in this disease. Since EBV infection is considered as an environmental trigger, it is one of the factors contributing to the pathogenesis of RA. As mentioned in the literature that EBV infection is widespread and 95% of all adults display serologic signs of previous infection, it is known that patients of RA have elevated levels of antibodies to latent and replicative EBV proteins and in particular to EBNA-1.[8–10] Anizilotti *et al*,[11] stated that antibodies specific for a deiminated VCP belonging to IgA and IgM isotype can be found in a few cases of RA. Anti-VCP IgA either alone or co-expressed with IgG or IgM are not associated with erosive or with active disease.

Rea *et al*.[12] states that acute illness was characterized by presence of VCA-IgG and VCA-IgM by ELISA and by absence of EBNA in most but not all patients. Costenbader and Karlson[13] points to a common virus such as EBV that could act as a trigger in genetically susceptible hosts. The EBV carrier state is characterized by latent infection of the general B cell pool, and by chronic virus replication in the Caucasian populations, most healthy carriers seem to harbor one dominant transforming virus strain usually of Type 1 rather than Type 2 and are detectable in the blood and in the throat. Patients with existing RA have higher levels of antibodies against several EBV-encoded proteins including VCA, EA, EBNA-1 and EBNA-2 than HC. The presence of RF does not seem to be related to these elevation and these are not influenced by age, duration of RA, disease activity or RA treatment. Patients with RA have significantly increased numbers of circulating EBV-infected B cells.

Blaschke *et al*,[14] also showed that EBV infection may be involved in the pathogenesis of RA. Pratesi *et al*,[15] have shown that sera from RA patients react with a deiminated protein encoded by EBV antibodies that are present exclusively in RA sera, which bind the citrullinated peptide corresponding to sequence 35–58 of EBNA-1 and recognize it in the context of the whole protein that bind to *in vivo* deiminated EBNA-1 These results suggest a role for EBV infection in the induction of disease-specific antibodies in RA. The discovery of the high specificity of antibodies to citrullinated proteins in RA provides insight into its cause. Recent advancements show that anti-citrullinated collagen type CII antibodies (CII)- directly interact with the citrullinated modification of the arginine side chain and that they are pathogenic, providing a good starting point to understand their role in the human disease and suggesting that they are citrullinated. CII might be involved in the immune self-perpetuation of arthritis in RA.[16] Whether increased levels of EBV in patients with RA are the cause or effect does not seem that this phenomenon is not related to latent viruses.[17] Even if the increased EBV in RA is due to the underlying genetic dysregulation in the immune response, the virus could have a significant role in RA joint disease in a number of different ways.[18] Similarly, Catyalano *et al*.[19] states that in both Normals and RA patients, there was significant association between the presence of antibodies to RA nuclear antigen and the titers of antibodies to EBV. These titers were equivalent to those of RA patients.

Therefore, from our studies and as published in the literature, we can say that there is a possible association of EBV and RA. An RA develops a strong humoral immune response to EBV nuclear antigen, which in part accounts for the increased titers of antibody to RA nuclear antigen. A new concept is being developed on the basis of sequence homology between the genetic RA susceptibility determinant HLADR4 and the EBV glycoprotein. Thus we may conclude that there is a production of ACPA response by RA patients, which is based on the EBNA-1 specific T cells and the anti-VCP antibody response is produced in early rheumatoid patients towards the deaminated proteins.
